The article "Assessment of Ecological Environment Quality for Urban Sustainable Development Based on AHP" was retracted in 2023. Reasons: unreliable results or conclusions; concerns about the data; concerns about the peer review; concerns about the citations.

# Assessment of Ecological Environment Quality for Urban Sustainable Development Based on AHP

**DOI:** 10.1155/2022/4056713

**Published:** 2022-09-01

**Authors:** Liang Zhou

**Affiliations:** School of Design and Art, Hunan Institute of Technology, Hengyang 421002, Hunan, China

## Abstract

Cities are gradually developed on the basis of adapting and transforming the natural environment. In a certain urban area, human activities, natural environment, and other factors and their mutual influence constitute the urban ecological environment. Therefore, the evaluation of urban ecological environment quality is of great significance to the analysis of urban development. This paper takes a city in Western China as the evaluation object, uses AHP to determine the index weight, reasonably analyzes the current situation of the urban ecological environment, and further comprehensively evaluates the quality of the urban ecological environment. The study shows that from 2013 to 2018, the comprehensive capacity of the city's ecological environment quality showed a steady upward trend, except that the natural disasters of floods and mudslides in 2014 had a certain degree of fluctuation. The comprehensive index of ecological environment quality has increased from 0.337 in 2013 to 0.412 in 2018. The overall level is still low, but the development speed is relatively stable. The urban ecological environment has been gradually improved, and society, economy, and nature have maintained a certain degree of sustainable development.

## 1. Introduction

The product of the development of human society to a certain stage has produced cities, so the emergence of cities is a symbol of human progress. In 1971, UNESCO put forward the concept of “eco city” in the man and biosphere plan, emphasizing the realization of a complex natural symbiosis system and sustainable development of social economy, and the creation of harmony between man and nature. However, the harmonious coexistence between man and nature has not been realized. On the contrary, the greenhouse effect, global warming, and other phenomena indicate that the Earth on which civilization depends is suffering damage. The current large-scale urbanization and urban modernization in China are facing severe ecological problems: first, the natural resources and the environment are severely damaged [1]. The city is an artificial system based on the natural environment. If this artificial system is in the process of establishment and development, inadequate treatment of nature and protection of nature can easily cause the original ecological environment in the urban area to gradually shrink and trigger a vicious ecological environment effect [2, 3]. The second is that the living resources are seriously polluted. The water pollution caused the shortage of water resources and air pollution has become a bottleneck in the development of many cities. The third is soil heavy metal pollution, which occupies more and more solid wastes [4–6]. With the continuous improvement of the output requirements of agricultural products per unit area, there are more and more chemical fertilizers and pesticides per unit of land, and more and more undecomposable substances remain in the soil. Once the soil is polluted, it is difficult to control because there are many elements of the urban ecological environment. An urban ecosystem is an open ecosystem with large capacity, multiflow, high density, and fast operation. The imperfect relationship network of the system and the intensity of various flows in the natural ecosystem make its decomposition function inadequate and its self-regulation and self-sustaining ability weak. Besides environmental pollution factors, many scholars also use the status of natural resource holdings and biodiversity to reflect the quality of the urban ecological environment [7, 8]. Broadly speaking, the quality of the urban ecological environment is a combination of the quality of the socio-economic environment and the quality of the city's natural environment. From this perspective, the quality of the urban ecological environment can include several aspects such as air quality, acoustic environmental quality, solid waste, soil environmental quality, and water environmental quality [9]. As the concept of sustainable development gradually gains popularity among the people, many countries regard sustainable development as the most important concept and principle when evaluating regional ecological quality and put forward a number of index systems that are conducive to the sustainable development of cities [10–12]. The so-called sustainable development capacity of the ecological environment is the dynamic identification of the total capacity of the regional environment. The human development of the region, the utilization of resources, and the transformation of nature should be maintained within the allowable capacity of the environment. In other words, only by maintaining the quality of the real environment within the allowable bearing standard can we seek more reasonable development. The sustainable development ability is the necessary guarantee for the smooth implementation of the sustainable development strategy. Specifically, sustainable development capacity involves decision-making, management, economy, resources, science and technology, human resources, and other aspects of a certain region. Local governments are the main force in implementing the sustainable development strategy. For example, in 1990, the United Nations Organization for Economic Cooperation and Development (OECD) launched a project to study ecological environment indicators and adopted the PSR system, which mainly represents the pressure caused by human activities on the ecological environment [13–15]. The United States Environmental Protection Agency, Washington Development and Research Office, and other units jointly conducted a comprehensive evaluation of the ecological health of Atlanta in the United States. They selected 32 indicators as the evaluation index system, including population per unit area, rate of population change, human utilization Index, road density index, annual deposition of nitrogen in a certain period of time, annual deposition of sulfur in a certain period of time, annual rate of change of ozone in a certain period of time, and the ratio of elements such as rivers and forests in urban areas [16–18].

The article "Assessment of Ecological Environment Quality for Urban Sustainable Development Based on AHP" was retracted in 2023. Reasons: unreliable results or conclusions; concerns about the data; concerns about the peer review; concerns about the citations.

The implementation of urban community planning and design in China inevitably requires saving resources and harmonious coexistence with nature, and the construction of ecological civilization is its due meaning. The basis for strengthening the construction of ecological civilization is to systematically understand the evaluation system and risk warning of ecological civilization construction. Only by establishing the evaluation system of ecological civilization construction as soon as possible can it play a due role in the management department's formulation of corresponding supervision strategies, the establishment of its key monitoring areas, the improvement of its ecological supervision efficiency, and the prevention of ecological risks. This article is based on ecological theory and sustainable development theory. This study takes a city in western China as an example and uses the analytic hierarchy process to establish an urban ecological environment quality evaluation index system to provide guidance for the analysis and evaluation of urban ecological environment quality.

The evaluation of urban ecological environment quality needs to be considered from both qualitative and quantitative aspects, analyze the factors affecting the urban ecological environment, understand the relationship between urban ecological environment quality and urban economic development and social stability, and comprehensively consider various factors in the evaluation of urban ecological environment construction, so as to better complete the evaluation and analysis of urban ecological environment quality.

## 2. Methods and Materials

### 2.1. AHP Model

Analytic hierarchy process (AHP) is a systematic method that takes a complex multiobjective decision-making problem as a system, decomposes the objective into multiple objectives or criteria, and then decomposes it into several levels of multiple indicators (or criteria and constraints), and calculates the single ranking (weight) and total ranking of the levels through the qualitative index fuzzy quantification method, so as to be the objective (multiobjective) and multischeme optimization decision-making. The basic principle of the analytic hierarchy process is to divide the basic elements of the scheme into layers and evaluate each layer separately. Each layer needs to make a judgment and comparison on the basis of the upper layer to finally form good calculation elements so that relevant weights and evaluation criteria can form the best evaluation scheme, and the derivation of the best scheme is carried out by means of weighted average.

The article "Assessment of Ecological Environment Quality for Urban Sustainable Development Based on AHP" was retracted in 2023. Reasons: unreliable results or conclusions; concerns about the data; concerns about the peer review; concerns about the citations.

The target layer is the comprehensive index of the ecological environment quality of the city. The subtarget layer includes social, economic, and natural indicators. The criterion layer includes population factors, social security, resource allocation, pollution control, industrial structure, economic income, air quality, acoustic environment quality, water environment quality, and biological environment quality [19]. Indicators include natural population growth rate, urbanization level, number of hospital beds per 10,000 people, education investment as a percentage of GDP, per capita housing area, urban population registered unemployment rate, industrial wastewater discharge compliance rate, the comprehensive utilization rate of industrial solid waste, harmless treatment rate of domestic waste, the proportion of tertiary industry in GDP, GDP growth rate, annual disposable income per capita, GDP per capita, urban-rural income ratio, smoke and dust control area coverage, urban air pollution index API, the average value of the environmental noise equivalent sound level in the urban area, the compliance rate of urban drinking water source water quality, the urban green coverage rate, and the urban per capita public green area. The analytic hierarchy process model is shown in Table 1.

### 2.2. Analytic Hierarchy Process Calculation

The judgment matrix between the target layer and the subtarget layer is shown in Table 2.

The judgment matrix between the subtarget layer and the criterion layer is shown in Table 3–5.

The weight of the index system is shown in Table 6.

### 2.3. Comprehensive Evaluation Calculation

This article shows the relevant data of a city in western China from 2013 to 2018. The analytic hierarchy process is used to calculate the weight of each indicator, and on this basis, the corresponding indicator values of each level in the city's urban ecological environment quality evaluation indicator system are calculated. Finally, the indicator value of the target layer is calculated, which is the final evaluation of the comprehensive index of urban ecological environment quality in this city.

The article "Assessment of Ecological Environment Quality for Urban Sustainable Development Based on AHP" was retracted in 2023. Reasons: unreliable results or conclusions; concerns about the data; concerns about the peer review; concerns about the citations.

#### 2.3.1. Calculation of the Evaluation Index at the Index Level

(1) $$\begin{array}{c} \text{When the index value is as large as possible},\;Di=\frac{Zi}{Si},\\ \text{When the index value is as small as possible},\;Di=\frac{Si}{Zi}. \end{array}$$

Here, *Di* is the evaluation index value of the *i*-th index, *Zi* is the data value of the *i*-th index, and *Si* is the standard value of the *i*-th index.

#### 2.3.2. Calculation of the Criterion-Level Evaluation Index

The criterion-level evaluation index is derived from the arithmetic average value of the evaluation index of the index-level indicators contained in the level, and its calculation formula is as follows:

(2) $$\begin{array}{c} Ci=\sum_{i=1}^{m}\frac{Di}{m}. \end{array}$$

Here, *Ci* is the evaluation index value of the *i*-th index, *m* is the number of index-level indexes included in the criterion level, and *Di* is the evaluation index value of the *i*-th index in the index level.

#### 2.3.3. Calculation of Subtarget Layer Index

The evaluation index of the subobjective level is obtained by multiplying the evaluation index of the criterion level index contained in it by their respective weights and summing them. The calculation formula is as follows:

(3) $$\begin{array}{c} Bi=\sum_{i=1}^{n}Ci\cdot Wi. \end{array}$$

Here, *Bi* is the evaluation index value of the *i*-th index, *n* is the number of criterion level index items included in the subobjective layer, *Ci* is the evaluation index value of the *i*-th index of the criterion level, and *Wi* is the weight of the *i*-th index of the criterion level.

#### 2.3.4. Calculation of the Target Layer Index

The comprehensive index of the target layer is based on the indexes of each layer and is added again according to their respective weights. The calculation formula is as follows:

(4) $$\begin{array}{c} A=\sum_{i=1}^{n}Bi\cdot Wi, \end{array}$$

where *A* is the comprehensive evaluation index value of the target layer, *n* is the number of subtarget layer index items included in the target layer, *Bi* is the evaluation index value of the *i*-th index of the subtarget layer, *Wi* is weight of the *i*-th index of the subtarget layer.

### 2.4. Evaluation Basis

The numerical value of the comprehensive index calculated according to the calculation does not actually have any image significance. It is necessary to classify and define the comprehensive index of urban ecological environment quality. In the grade standard, the suitability index is equal to 0.65 as the passing line. The larger the value, the higher the suitability grade. It also shows that the quality of the urban ecological environment is better, and the sustainable development is stronger. Conversely, the smaller the value, the lower the suitability level, and it also indicates that the quality of the urban ecological environment is worse, and the sustainable development is weaker (Table 7).

The article "Assessment of Ecological Environment Quality for Urban Sustainable Development Based on AHP" was retracted in 2023. Reasons: unreliable results or conclusions; concerns about the data; concerns about the peer review; concerns about the citations.

## 3. Result

### 3.1. Analysis of Comprehensive Index of Ecological Environment Quality

From 2013 to 2018, the comprehensive capacity of the city's ecological environment quality generally showed a steady increase. Except for the summer floods and mudslides in 2014, social indicators, economic indicators, and natural indicators all fluctuate to varying degrees, as shown in Figure 1. From the perspective of the comprehensive index of ecological environment quality, it has developed from 0.337 in 2013 to 0.412 in 2018. The overall level is still low, but the development speed is relatively stable. From the perspective of the index classification, the urban ecological environment has been upgraded from level 4 in 2013 to level 3 in 2018. Most of the indicators have developed to a certain extent, indicating that the city's ecological environmental quality is gradually improving.

In the overall environmental development of the city, the overall development of the social environment is relatively stable. The population growth has been effectively controlled, various social infrastructure construction has been gradually improved, the unemployment rate has been drastically reduced, and pollution control has achieved certain results. The overall economic environment is developing slowly. Due to summer floods and mudslides in 2014, the city actively promoted economic system reforms and industrial restructuring which greatly improved people's living standards. The natural environment has developed relatively rapidly. Due to the impact of natural disasters, the natural ecological environment has been severely damaged. However, with the active advancement of postdisaster reconstruction work, the ecological restoration of the natural environment has developed rapidly, especially in the greening construction.

### 3.2. Analysis of the Comprehensive Index of Social Environment

During the period from 2013 to 2018, the overall social and environmental quality index of the city showed a steady development trend. The social and environmental infrastructure was continuously improved, and the living standards of the people continued to improve. However, the overall development of the social environment was still slow, as shown in Figure 2.

The article "Assessment of Ecological Environment Quality for Urban Sustainable Development Based on AHP" was retracted in 2023. Reasons: unreliable results or conclusions; concerns about the data; concerns about the peer review; concerns about the citations.

In 2013 and 2018, the city's natural population growth rate remained negative, while the population growth rate in 2018 has risen to 1.2%. The population has increased year by year, but the overall growth rate is controlled within a reasonable range. The level of urbanization is still lower than the standard value of 70% in moderately developed countries. The population is the main body of the urban ecological environment. Too much denseness will cause pressure on space and the environment [20].

The social public infrastructure is continuously developed and improved, but the overall level still has a certain gap with the standards of the moderately developed countries. The proportion of education investment has increased relatively, but the overall level is still lower than the corresponding standard level [21]. In 2018, the city's per capita housing area reached 36.1 square meters, far higher than the standard value of 16 square meters, and the unemployment rate dropped from 2.4% in 2013 to 0.27% in 2018. The quality of life of the people has improved. In recent years, due to the needs of urban development, the accelerated development of industrial industries has caused certain damage to the urban environment. Environmental protection has received more and more attention. The city has increased its pollution control efforts, vigorously rectified environmental pollution problems, and implemented corresponding measures for related enterprises. Corrective measures have been taken and some results have been achieved [22].

### 3.3. Analysis of Comprehensive Index of Economic Environment

From 2013 to 2018, the overall economic and environmental quality index of the city showed a steady and slow development trend. In 2014, due to the impact of natural disasters, the overall economic and environmental level dropped to the level equivalent to two years ago, as shown in Figure 3. The impact of natural disasters on the environment is measured by the following five indicators: (1) direct economic losses caused by geological disasters; (2) investment in geological disaster prevention and control; (3) direct economic loss caused by forest fire; (4) comprehensive control rate of forest diseases, pests, and rodents; (5) direct economic loss caused by environmental pollution and destruction. With the progress of postdisaster reconstruction, the economic environment has gradually recovered and developed, but the overall level has not improved much.

Due to the impact of natural disasters in 2014, the city's economic development was hit hard, the overall level dropped sharply, the city's industrial structure was severely damaged, and the GDP growth rate in the same year showed negative growth. From the analysis of the major natural disasters that have occurred to human beings, it shows that the direct loss of natural disasters does not have a significant impact on the national economy. General natural disasters have an impact in the short term, and it is difficult to constitute a fundamental disturbance to the huge capital market of the whole country. Since then, until 2018, various economic indicators have gradually recovered, but the development speed has remained slow. Per capita GDP exceeded the standard value for the first time in 2017, and increased significantly in the subsequent period, reaching 48,518 yuan in 2018. In 2017, the annual per capita disposable income reached the relative standard value requirement and exceeded a certain level in 2018. The development trend is good, marking the great improvement and improvement of the quality of life of the people. There is still a certain gap in the urban-rural income ratio, which is related to the low degree of urbanization and the excessive density of the rural population [23].

The article "Assessment of Ecological Environment Quality for Urban Sustainable Development Based on AHP" was retracted in 2023. Reasons: unreliable results or conclusions; concerns about the data; concerns about the peer review; concerns about the citations.

### 3.4. Analysis of the Comprehensive Index of Natural Environment

From 2013 to 2018, the city's natural environmental quality comprehensive index showed an upward trend year by year, as shown in Figure 4. However, due to the impact of summer floods and mudslides in 2014, the urban natural environment was severely damaged, the structure of the ecosystem was changed, and the function of the ecosystem was greatly affected.

Before the floods and mudslide disasters, the city's socio-economic development was stable, and the trend was good. Financial revenue has increased steadily, the people's income has increased rapidly, and the quality of life has improved rapidly. The industrial economy has developed rapidly, the scale of investment in the city has continued to expand, and the overall level of urban prices has been relatively stable. After the natural disaster, the social economy was severely damaged, especially the secondary industry suffered huge losses. The total agricultural production decreased, and the main crops were affected by the dual impact of floods and mudslides. Large-scale collapses, landslides, and corresponding formation of mud-rock flows and dammed lakes have been caused in the mountainous area, and the natural ecological environment has been severely damaged [24]. Animal habitats, rare animals and plants, native vegetation, and the living environment of wild animals and plants have all been severely affected, the structure of the ecosystem has changed, and the function of the ecosystem has been damaged.

The article "Assessment of Ecological Environment Quality for Urban Sustainable Development Based on AHP" was retracted in 2023. Reasons: unreliable results or conclusions; concerns about the data; concerns about the peer review; concerns about the citations.

### 3.5. Urban Development Suggestions

It is necessary to promote urban ecological environment protection through scientific and technological innovation, and vigorously research, develop and promote key applicable technologies for urban environmental protection in the main urban areas. We should fully publicize environmental awareness to the public, give full play to the role of news media and social organizations, strengthen public publicity through various media, and popularize relevant policies and regulations on ecological and environmental protection. And, let the masses imperceptibly contact and accept the correct environmental protection awareness and concepts in their daily life and consciously participate in the actual actions of environmental protection.

## 4. Conclusion

Cities are gradually developed on the basis of adapting and transforming the natural environment. In a certain urban area, human activities, natural environment, and other factors and their mutual influence constitute the urban ecological environment. Therefore, the evaluation of urban ecological environment quality is of great significance to the analysis of urban development.

1. This paper chooses to use the analytic hierarchy process to determine the index weights. After calculation, the comprehensive index of the ecological environment quality of a city in western China has developed from 0.337 in 2013 to 0.412 in 2018, indicating that the urban ecological environment of this city has changed from 2013 to 2018. The current ecological environment quality of the city is average, and the economy, society, and environment are not yet in harmony. From the perspective of index classification, the ecological environment of the city has been upgraded from the level 4 standard in 2013 to the level 3 standard in 2018. The overall level is still low, but the urban ecological environment is gradually improving, maintaining a certain degree of sustainability.
2. During the period from 2013 to 2018, the comprehensive capacity of the ecological environment of a city in western China generally showed a steady increase, except for the impact of floods and mudslides in 2014. The overall level of the comprehensive index of ecological environment quality is still low, but the development speed is relatively stable. The overall development of the social environment is relatively stable, the overall economic environment develops slowly, and the natural environment develops relatively rapidly. Although affected by the natural disasters in 2014, due to the active advancement of postdisaster reconstruction, the ecological restoration of the natural environment has developed rapidly, and the urban environment has been improved. [25, 26].

The article "Assessment of Ecological Environment Quality for Urban Sustainable Development Based on AHP" was retracted in 2023. Reasons: unreliable results or conclusions; concerns about the data; concerns about the peer review; concerns about the citations.

## Figures and Tables

**Figure 1:** Change curve of a comprehensive index of ecological environment quality.

**Figure 2:** The change curve of the comprehensive index of social environmental quality.

**Figure 3:** The change curve of the comprehensive index of social environmental quality.

**Figure 4:** The change curve of the comprehensive index of natural environmental quality.

**Table 1:** The analytic hierarchy process model of urban ecological environment quality evaluation.

Target layer	Subtarget layer	Criterion layer	Index layer
Comprehensive index of ecological environment quality, A	Natural indicators, B3	Biological environment quality, C10	Per capita public green area, D20
			Urban green coverage rate, D19
		Water environmental quality, C9	Drinking water source water quality compliance rate, D18
		Acoustic environmental quality, C8	Average value of environmental noise equivalent sound level, D17
		Air quality, C7	Air pollution index, D16
			Coverage rate of smoke and dust control area, D15
	Economic indicators, B2	Economic income, C6	Urban-rural income ratio, D14
			GDP per capita, D13
			Annual disposable income per capita, D12
		Industrial structure, C5	GDP growth rate, D11
			The proportion of tertiary industry in GDP, D10
	Social indicators, B1	Pollution control, C4	Harmless treatment rate of domestic garbage, D9
			Comprehensive utilization rate of industrial solid waste, D8
			Industrial wastewater discharge compliance rate, D7
		Resource allocation, C3	Registered unemployment rate of urban population, D6
			Housing area per capita, D5
		Social security, C2	Education investment as a proportion of GDP, D4
			Number of hospital beds per 10,000 people, D3
		Demographic factors, C1	Urbanization level, D2
			Natural population growth rate, D1

**Table 2:** Judgment matrix between the target layer and the subtarget layer.

Comprehensive index of ecological environment quality, A	Social indicators, B1	Economic indicators, B2	Natural index, B3
Social indicators, B1	1	1	1/3
Economic indicators, B2	1	1	1/3
Natural index, B3	3	3	1

CI: RI < 0.1, with satisfactory consistency.

**Table 3:** Judgment matrix of three indicators of a social environment.

Social environmental indicators, B1	Demographic factors, C1	Social security, C2	Resource allocation, C3	Pollution control, C4
Demographic factors, C1	1	1/5	1/3	1/5
Social security, C2	5	1	1	1/3
Resource allocation, C3	3	1	1	1/3
Pollution control, C4	5	3	3	1

CI: RI < 0.1, with satisfactory consistency.

**Table 4:** Judgment matrix of two indicators of the economic environment.

Economic and environmental indicators, B2	Industrial structure, C5	Economic income, C6
Industrial structure, C5	1	1
Economic income, C6	1	1

CI: RI < 0.1, with satisfactory consistency.

The article "Assessment of Ecological Environment Quality for Urban Sustainable Development Based on AHP" was retracted in 2023. Reasons: unreliable results or conclusions; concerns about the data; concerns about the peer review; concerns about the citations.

**Table 5:** Judgment matrix of two indicators of the natural environment.

Natural indicators, B3	Air quality, C7	Acoustic environmental quality, C8	Water environmental quality, C9	Biological environment quality, C10
Air quality, C7	1	3	1/7	1/5
Acoustic environmental quality, C8	1/3	1	1/9	1/7
Water environmental quality, C9	7	9	1	1/3
Biological environment quality, C10	5	7	3	1

CI: RI < 0.1, with satisfactory consistency.

**Table 6:** Index system weight.

Subtarget layer		Criterion layer		Index layer	
Indicator	Weight	Indicator	Weight	Indicator	Weight
Natural indicators, B3	0.6	Biological environment quality, C10	0.312	Per capita public green area, D20	0.156
				Urban green coverage rate, D19	0.156
		Water environmental quality, C9	0.209	Drinking water source water quality compliance rate, D18	0.209
		Acoustic environmental quality, C8	0.026	Average value of environmental noise equivalent sound level, D17	0.026
		Air quality, C7	0.053	Air pollution index, D16	0.027
				Coverage rate of smoke and dust control area, D15	0.027

Economic indicators, B2	0.2	Economic income, C6	0.1	Urban-rural income ratio, D14	0.018
				GDP per capita, D13	0.037
				Annual disposable income per capita, D12	0.045
		Industrial structure, C5	0.1	GDP growth rate, D11	0.025
				The proportion of tertiary industry in GDP, D10	0.075

Social indicators, B1	0.2	Pollution control, C4	0.102	Harmless treatment rate of domestic garbage, D9	0.034
				Comprehensive utilization rate of industrial solid waste, D8	0.034
				Industrial wastewater discharge compliance rate, D7	0.034
		Resource allocation, C3	0.039	Registered unemployment rate of urban population, D6	0.007
				Housing area per capita, D5	0.032
		Social security, C2	0.045	Education investment as a proportion of GDP, D4	0.034
				Number of hospital beds per 10,000 people, D3	0.011
		Demographic factors, C1	0.013	Urbanization level, D2	0.002
				Natural population growth rate, D1	0.011

**Table 7:** Classification of a comprehensive index of urban ecological environment quality.

Level	Comprehensive index	Comments
1	≥0.8	Strong sustainable development
2	0.65∼0.8	Medium sustainable development
3	0.35∼0.65	Weak sustainable development
4	0.20∼0.35	Sustainable development is hindered
5	≤0.2	Sustainable development is severely hindered

## Data Availability

The figures and tables used to support the findings of this study are included in the article.
